This article has been retracted.

# Effects of Dydrogesterone Tablets Combined with Zishen Yutai Pills on Threatened Abortion in Early Pregnancy and Pregnancy Outcomes

**DOI:** 10.1155/2022/4593637

**Published:** 2022-07-19

**Authors:** Xuehong Chen, Xiaoxiao Qiu, Yaojuan Jin

**Affiliations:** ^1^Department of Obstetrics and Gynecology, Linhai Second People's Hospital, Linhai, 317016 Zhejiang, China; ^2^Department of Obstetrics and Gynecology, Taizhou Municipal Hospital, Taizhou, 318000 Zhejiang, China

## Abstract

**Objective:**

To explore the effect of dydrogesterone tablets combined with Zishen Yutai pills on threatened abortion in early pregnancy and pregnancy outcomes.

**Methods:**

This study retrospectively analyzed the clinical data of 100 patients with threatened abortion in early pregnancy who came to the Linhai Second People's Hospital/Taizhou Municipal Hospital from January 13, 2021, to January 13, 2022. According to different treatment methods, 48 patients treated with progesterone injection were assigned to the control group (CG), while 52 cases with the combined therapy of dydrogesterone tablets and Zishen Yutai pills were assigned to the observation group (OG). The two groups were compared in terms of the following parameters: treatment efficacy, whole blood high shear viscosity, hematocrit (HCT), plasma fibrinogen (FIB) level, spiral artery pulsatility index (PI), uterine spiral artery blood flow resistance index (RI), lumbar and abdominal pain relief time, hemostasis time, estrogen levels, pregnancy outcomes, neonatal adverse outcomes, and incidence of adverse reactions.

**Results:**

Compared with CG, the therapeutic effect in OG was observed to be evidently better, and its pain relief time and hemostasis time in the waist and abdomen were markedly shorter. After treatment, the whole blood high shear viscosity, FIB, RI, PI, and estrogen levels of both groups improved statistically compared with those before treatment, with more significant improvements in OG compared with CG. OG was also superior to CG with markedly lower incidence of preterm birth, miscarriage, neonatal adverse outcomes, and adverse reactions and a drastically higher full-term pregnancy rate.

**Conclusion:**

Zishen Yutai pill combined with dydrogesterone tablets is of remarkable therapeutic effect in treatment of early threatened abortion, which can significantly improve clinical symptoms and pregnancy outcomes of patients, with a high safety profile, which is worthy of clinical application.

## 1. Introduction

Threatened abortion refers to a condition in which signs of miscarriage such as vaginal bleeding and paroxysmal lower abdominal pain occur before 28 weeks of pregnancy, but with no obvious abnormality in pelvic examination or discharge of pregnancy products and a size of the uterus consistent with the pregnancy cycle [1]. If the patient's symptoms persist and worsen, there is an inevitable risk of progressing into a complete miscarriage [2]. Threatened abortion occurs in 20% of all pregnancies and is diagnosed when vaginal bleeding with or without abdominal pain occurs during the first half of pregnancy [3]. Early threatened abortion refers to the symptoms of threatened abortion within 1-12th weeks of pregnancy, with some patients experiencing early pregnancy reactions such as fatigue, lethargy, fatigue, loss of appetite, nausea, and vomiting [4]. Prompt miscarriage treatment can prevent inevitable miscarriage, and supplementation of progesterone, human chorionic gonadotropin (hCG), and immunotherapy also have certain effects but are barely satisfactory [5].

Western medicine believes that the occurrence of threatened abortion is related to factors such as heredity, immunity, endocrine, infection, endometrial function, and reproductive tract abnormalities, among which endocrine abnormalities are the common cause. Therefore, supplementing hormones necessary during pregnancy is a common clinical treatment [6]. Dydrogesterone is a natural progesterone extracted from tubers with a chemical structure highly similar to progesterone. Oral administration is highly biologically active, almost binding exclusively to progesterone receptors and showing highly selective progesterone action [7, 8]. However, Traditional Chinese Medicine (TCM) believes that threatened abortion is caused by insufficient Qi in the spleen and stomach metaplasia, as well as insufficiency of both the spleen and the kidney. It belongs to the categories of “uneasy fetal movement” and “fetal leakage,” the best solution to which is to nourish Qi and tonic and strengthen the spleen and kidney [9]. Zishen Yutai pill is an empirical formula for the prevention and treatment of threatened abortion. In this formula, dodder, mulberry, Atractylodes, Eucommia, and Tatsuya are used in combination to nourish the liver and kidney, as well as Qi and Yuan. Ginseng, Rehmannia glutinosa, and Polygonum multiflorum can invigorate the spleen and Qi, nourish blood, and soothe miscarriage [10].

Integrating traditional Chinese and Western medicine is a characteristic treatment plan in China. However, few studies have analyzed the efficacy of dydrogesterone tablets combined with Zishen Yutai pills in the treatment of early threatened abortion. We took this as a breakthrough in our study and analyzed its effect on the curative efficacy and pregnancy outcome of patients with threatened abortion in early pregnancy. We believe that this study can not only provide more reference treatment options for such patients but also further promote the development of integrated Chinese and Western medicine.

## 2. Materials and Methods

### 2.1. Clinical Information

We retrospectively analyzed the clinical data of 100 patients with threatened abortion in early pregnancy who came to the Linhai Second People's Hospital/Taizhou Municipal Hospital from January 13, 2021, to January 13, 2022. According to different treatments they received, patients (average age: 27.21 ± 2.36 years) were divided into the following two groups: a control group (CG; *n* = 48) treated with progesterone injection and an observation group (OG; *n* = 52) treated by dydrogesterone tablets combined with Zishen Yutai pills. Inclusion criteria are as follows: (1) positive urine HCG examination, (2) presence of symptoms such as vaginal bleeding and abdominal pain, (3) normal intrauterine embryos by color Doppler ultrasonography, and (4) no excretion of pregnancy material. Exclusion criteria are as follows: (1) allergic to the drugs used in this study; (2) vaginal bleeding caused by other intrauterine diseases such as placenta previa and hydatidiform mole; (3) uterine and/or ovarian tumors, genital tract malformations, or other serious systemic diseases; (4) severe cognitive impairment, mental illness, or obvious memory impairment; and (5) poor medication compliance. With approval from the Ethics Committee, this research also complies with the Declaration of Helsinki, with all patients provided the written informed consent concerning their agreement for participation.

### 2.2. Treatment Methods

Pregnant women in CG were treated with intramuscular injection of 20 mg progesterone (Zhejiang Xianju Pharmaceutical Co., Ltd., approved by National Medicine H33020828), once daily. Those in OG were given Zishen Yutai pills (Guangzhou Baiyunshan Zhongyi Pharmaceutical Co., Ltd., Z44020008) 5 g once, 3 times a day, as well as dydrogesterone tablets (Abbott Trading Co., Ltd., Imported Drug Registration Certificate No. H20130110/H20170221) that was administrated 3 times a day orally with the loading dose of 40 mg and then 10 mg once. During the period, the dosage can be adjusted according to each patient's condition. All patients were treated for 2 consecutive weeks.

### 2.3. Outcome Measures

(1) Therapeutic effects of the two groups were evaluated and compared based on color Doppler ultrasound results, with evaluation criteria as follows: cured: the fetal heart beat was normal, with the size of the uterus, embryonic development, etc. consistent with the pregnancy cycle, and disappearance of symptoms such as vaginal bleeding, abdominal pain, and low back pain; markedly effective: no obvious abnormality, nor symptoms such as vaginal bleeding, with markedly relieved abdominal and low back pain; effective: all items are basically consistent with the pregnancy cycle, and symptoms such as vaginal bleeding, abdominal pain, and low back pain are improved; and ineffective: the size of the uterus does not match the pregnancy cycle, the embryonic development is defective or stopped, and symptoms such as vaginal bleeding, abdominal pain, and low back pain are not improved or even worsened. Total effective rate of treatment = (number of cured cases + number of markedly effective cases)/total number of cases × 100%. (2) Hematocrit (HCT), whole blood high shear viscosity, and plasma fibrinogen (FIB) levels before and after treatment were detected and compared between the two groups. (3) Color Doppler was used to detect and compare spiral artery pulsatility index (PI) and uterine spiral artery blood flow resistance index (RI) before and after treatment between the two groups. (4) Pain relief time and hemostasis time were also recorded and compared. (5) Estrogen levels, including serum progesterone (progesterone, P), estradiol (estradiol, E_2_), and human hCG levels, were measured before and after treatment using the enzyme-linked immunosorbent assay (ELISA) and compared between the two groups. (6) The pregnancy outcomes (preterm birth, miscarriage, and full-term pregnancy) were recorded and compared. (7) Adverse neonatal outcomes, including macrosomia, deformity, respiratory distress, and term low birth weight, were recorded and compared. (8) Incidence of adverse reactions during treatment were recorded and compared in two groups, including pruritus, erythema, and temporary vaginal bleeding. All patients were given symptomatic treatment when adverse reactions occurred.

### 2.4. Statistical Methods

Statistical analysis of data was conducted with SPSS 19.0 (IBM). The enumeration data were expressed as the number of cases/percentage (*n*/%) and analyzed using the *χ*^2^ test. The measurement data was recorded as mean ± standard deviation, and the intergroup comparison, intragroup comparison before and after treatment, and post hoc test were performed using the Student *t* test, paired *t* test, and LSD/*t* test, respectively. The significance level was *P* < 0.05.

## 3. Results

### 3.1. General Data Comparison

The two groups were comparable due to insignificant differences observed regarding age, body mass index (BMI), gestation, and other general data (*P* > 0.05, Table 1).

### 3.2. Comparison of Therapeutic Effects between Two Groups of Patients

The numbers of OG patients who were cured, treated markedly effective, effective, and ineffective after treatment were 35, 10, 5, and 2, respectively. Corresponding data of CG were 21, 12, 10, and 5, respectively, showing a significantly lower treatment effective rate than OG (*P* < 0.05, Table 2).

### 3.3. Comparison of Changes in Whole Blood High Shear Viscosity, HCT, and FIB Levels before and after Treatment between Two Groups

Before treatment, there was no marked difference in levels of whole blood high shear viscosity, HCT, and FIB between the two groups (*P* > 0.05). After treatment, there was no significant difference in HCT levels between the two groups, but the whole blood high shear viscosity and FIB were significantly lower than those before treatment, and the degree of decline in OG was significantly better than that in CG (*P* < 0.05, Figure 1).

### 3.4. Comparison of RI and PI before and after Treatment between Two Groups

Before treatment, OG and CG showed no marked difference in RI and PI (*P* > 0.05), while after treatment, RI and PI of both groups reduced statistically, and the degree of decline in OG was more evident compared with CG (*P* < 0.05, Figure 2).

### 3.5. Comparison of Pain Relief Time and Hemostasis Time between Two Groups

Abdominal pain relief time and hemostasis time of patients in OG were 4.11 ± 0.26 d and 4.22 ± 0.22 d, respectively, and those in CG were 6.56 ± 0.45 d and 5.4 ± 0.33 d, respectively. Pain relief time and hemostasis time of OG were comparatively and markedly shorter compared with CG (*P* < 0.05, Table 3).

### 3.6. Comparison of Progesterone Levels before and after Treatment between Two Groups

No significant difference was observed in levels of P, E2, and hCG between the two groups before treatment (*P* > 0.05), while their levels in both groups increased statistically after treatment and were higher OG compared with CG (*P* < 0.05, Figure 3).

### 3.7. Comparison of Pregnancy Outcomes between Two Groups of Patients

Rates of preterm birth, miscarriage, and full-term pregnancy in OG were 9.62%, 3.85%, and 86.54%, respectively, and those of CG were 25.00%, 16.67%, and 58.33%, respectively, indicating markedly higher rates of preterm birth and abortion and lower full-term pregnancy rate in CG compared with OG (*P* < 0.05, Table 4).

### 3.8. Comparison of Neonatal Outcomes between Two Groups of Patients

In OG, the numbers of neonates with macrosomia, deformity, respiratory distress, and term infants with low birth weight were 2, 1, 0, and 1, respectively, with the incidence of adverse outcomes of 7.69%. While those in CG were reported as 3, 4, 4, and 4, respectively, and the occurrence of adverse outcome was 31.25%, an incidence statistically higher than that of OG (*P* < 0.05, Table 5).

### 3.9. Comparison of Incidence of Adverse Reactions between Two Groups

After treatment, the number of patients with itching, erythema, and temporary vaginal bleeding in OG was 1, 1, and 0, respectively. And those in CG were 2, 3, and 3, respectively, showing a much higher incidence of adverse reaction compared with OG (*P* < 0.05, 16.67% vs. 3.85%, Table 6).

## 4. Discussion

Threatened abortion is common in obstetrics and gynecology, the etiology of which is complex and related to various factors such as maternal genetics, corpus luteum function, endocrine disorders, and environmental inducements [11]. It mostly occurs in early pregnancy and is closely related to luteal insufficiency, accounting for about 30% of spontaneous abortions [12]. Western medicine mostly uses progesterone supplementation to treat pregnant women with threatened abortion. Dydrogesterone tablets are commonly used clinically to supplement progesterone, which can promote the secretion of chorionic gonadotropin and endogenous progesterone, increase the endocrine activity of placental trophoblast, reduce the level of oxytocin, and antagonize the stimulation of uterus by prostaglandins, thus inhibiting uterine contractions and maintaining pregnancy [13, 14]. Some scholars have reported that oral dydrogesterone is effective in the treatment of threatened abortion with a low abortion rate and no congenital malformation [15]. However, results of related studies also showed that simple supplementation of hormones for threatened abortion in early pregnancy has certain but unsatisfactory effects [16].

According to TCM theory, threatened abortion belongs to the categories of “fetal leakage,” “uneasy fetal movement,” and “abdominal pain during pregnancy.” The disease is attributed to the insufficiency of both the spleen and the kidney and the debility of Chong and Ren channels. Therefore, in TCM clinics, the treatment guidelines for threatened abortion are tonifying the kidney and spleen, nourishing the blood to soothe miscarriage, and nourishing the Qi and the vitality [17]. In this study, Zishen Yutai pills combined with dydrogesterone tablets were used in the treatment of early threatened abortion. The results showed significantly better therapeutic effects in OG treated with combined medicine, with statistically shorter abdominal pain relief time and hemostasis time compared with CG. Past studies have also confirmed that TCM combined with dydrogesterone tablets is highly effective in early threatened abortion treatment, which can quickly and effectively stop bleeding, improve clinical symptoms, and increase the levels of progesterone and *β*-hCG in the body [18], consistent with our observation. Zishen Yutai pill is a famous prescription for the prevention and treatment of threatened abortion. In this formula, dodder, mulberry, Atractylodes Rhizoma, Eucommia ulmoides, and Ticrup are used together to nourish the liver and kidneys, Qi, and Yuan; ginseng, Rehmannia glutinosa, and Polygonum multiflorum are used to invigorate the spleen and Qi and nourish the blood to relieve miscarriage [19]. Modern research has also confirmed that Zishen Yutai pills can promote ovarian hormone secretion, ovulation, ovarian function, and uterine growth and development as well [20].

In normal pregnancy, maternal plasma volume increases by about 40% to meet the needs of uteroplacental perfusion. With the expansion and thickening of maternal peripheral vascular lumen, vascular resistance decreases, microcirculation blood flow increases, and blood viscosity decreases [21]. However, the increased maternal blood viscosity, in a state of hypercoagulation, can lead to reduced uteroplacental blood oxygen supply and insufficient perfusion, resulting in different degrees of poor pregnancy [22]. This study evaluated the effect of Zishen Yutai pills combined with dydrogesterone tablets on blood hypercoagulation and uteroplacental perfusion in patients with early threatened abortion. The results indicated that the high shear whole blood viscosity and FIB of both groups after treatment went markedly lower than those before treatment, but HCT did not fluctuate much. And after treatment, the high shear whole blood viscosity and FIB in OG were statistically lower compared with CG, suggesting that Zishen Yutai pills combined with dydrogesterone tablets may reduce the level of FBG, thereby reducing whole blood viscosity and blood hypercoagulability, increasing the uteroplacental blood oxygen supply, relieving hypoperfusion, and inhibiting the occurrence or deterioration of pathological pregnancy. This is also the first time we have observed that Zishen Yutai pills combined with dydrogesterone tablets could effectively improve blood viscosity and placental blood supply in patients with early threatened abortion.

In addition, this study revealed that RI and PI of both groups of patients decreased after treatment, and the decrease in OG was more significant, suggesting that Zishen Yutai pills combined with dydrogesterone tablets may reduce uterine artery blood flow and improve uteroplacental blood perfusion by reducing uterine arterial blood flow resistance, increasing uteroplacental blood flow, facilitating trophoblast infiltration into the placental bed and uterine spiral artery muscle layer normally, and providing nutritional support and environmental optimization for embryos, which are conducive to the normal development of embryos. Deficiency of estrogen and progesterone is also an important factor leading to threatened abortion [23]. Research [24] has shown that P, as a progesterone, can inhibit uterine contractions, promote the development of the reproductive system, and maintain the continuation of pregnancy; hCG can promote the generation of P in the first trimester, promote the body to secrete estrogen, and reduce the level of oxytocin to inhibit uterine contractions, thus preventing the occurrence of miscarriage; E2 is an estrogen secreted by P that can promote endometrial hyperplasia. Therefore, the lower levels of the above three may indicate that the body has the risk of miscarriage. This study showed that levels of serum P, E2, and hCG in both groups went significantly higher after treatment, with more obvious increase in OG, suggesting that Zishen Yutai pills combined with dydrogesterone tablets can effectively improve estrogen levels. Finally, pregnancy outcomes and adverse reactions were analyzed in two groups, and the results indicated that OG, compared with CG, had lower rates of abortion, adverse neonatal outcomes, and preterm birth and a higher term pregnancy rate. In addition, the incidence of adverse reactions in OG was comparatively and markedly lower, suggesting that Zishen Yutai pills combined with dydrogesterone tablets can effectively improve pregnancy outcomes of patients with early threatened abortion, with fewer adverse reactions and higher safety. Previous studies have pointed out that dydrogesterone can increase the pregnancy success rate of threatened abortion by improving body hormone levels, which is also consistent with our observation [25].

## 5. Conclusion

In conclusion, Zishen Yutai pill combined with dydrogesterone tablets has a significant therapeutic effect on early threatened abortion and can significantly improve the clinical symptoms of patients, possibly by improving blood rheology and uteroplacental perfusion. In addition, it can significantly improve the pregnancy outcomes of patients with a high safety profile, which is worthy of clinical application. However, this study has certain limitations. First of all, in the integration of traditional Chinese and Western medicine, there are other Chinese patent medicines in addition to Zishen Yutai pills, so further investigation is warranted to see whether there is a difference in clinical efficacy between the combined treatment of dydrogesterone tablets with other Chinese patent medicines and the combination drug therapy used in this study. Second, due to the small sample size, the conclusions we obtained still need to be demonstrated by subsequent expansion of sample size. We will further carry out multicenter clinical research with a larger sample in the future, so as to provide more data support for the treatment of patients with early threatened abortion.

## Figures and Tables

**Figure 1:** Comparison of changes of whole blood high shear viscosity, HCT, and FIB levels before and after treatment between two groups. (a) Comparison of whole blood high shear viscosity of two groups. (b) Comparison of HCT of two groups. (c) Comparison of FIB in two groups. ∗ indicates *P* < 0.05.

**Figure 2:** Comparison of RI and PI before and after treatment between two groups. (a) RI comparison of two groups. (b) PI comparison of two groups. ∗ means *P* < 0.05 when the two groups are compared.

**Figure 3:** Comparison of progesterone levels between two groups before and after treatment. (a) P comparison in two groups. (b) E2 comparison in two groups. (c) hCG comparison of two groups of patients. ∗ indicates *P* < 0.05.

**Table 1:** Comparison of general data.

Factors	Observation group *n* = 52	Control group *n* = 48	*t*/*χ*^2^	*P*
Age (years)	27.19 ± 2.16	27.23 ± 2.59	0.078	0.938
BMI (kg/m^2^)			0.004	0.948
≤23	30 (57.69)	28 (58.33)		
>23	22 (42.31)	20 (41.67)		
Gestation (days)	6.99 ± 0.47	7.1 ± 0.45	1.193	0.236
Gravida			0.051	0.822
≤1	40 (76.92)	36 (75.00)		
>2	12 (23.08)	12 (25.00)		
Vaginal bleeding time (d)			0.043	0.835
≤3	26 (50.00)	25 (52.08)		
>3	26 (50.00)	23 (47.92)		
Times of abortion			0.004	0.951
≤1	42 (80.77)	39 (81.25)		
>2	10 (19.23)	9 (18.75)		

**Table 2:** Comparison of therapeutic effect between two groups of patients.

Therapeutic effect	Observation group *n* = 52	Control group *n* = 48	*χ* ^2^	*P*
Cured	35 (67.31)	21 (43.75)	—	—
Markedly effective	10 (19.23)	12 (25.00)	—	—
Effective	5 (9.62)	10 (20.83)	—	—
Ineffective	2 (3.85)	5 (10.42)	—	—
Treatment effective rate	45 (86.54)	33 (68.75)	4.603	0.032

**Table 3:** Comparison of pain relief time and hemostasis time between two groups of patients.

Items	Observation group *n* = 52	Control group *n* = 48	*t*	*P*
Abdominal pain relief time (d)	4.11 ± 0.26	6.56 ± 0.45	33.65	<0.001
Hemostasis time (d)	4.22 ± 0.22	5.4 ± 0.33	21.19	<0.001

**Table 4:** Comparison of pregnancy outcomes between two groups.

Items	Observation group *n* = 52	Control group *n* = 48	*χ* ^2^	*P*
Preterm birth rate	5 (9.62)	12 (25.00)	4.187	0.041
Miscarriage rate	2 (3.85)	8 (16.67)	4.558	0.033
Full-term pregnancy rate	45 (86.54)	28 (58.33)	10.07	0.002

**Table 5:** Comparison of neonatal outcomes between two groups of patients (*n* (%)).

Adverse reactions	Observation group *n* = 52	Control group *n* = 48	*χ* ^2^	*P*
Fetal macrosomia	2 (3.85)	3 (6.25)	—	—
Deformity	1 (1.92)	4 (8.33)	—	—
Respiratory distress	0	4 (8.33)	—	—
Term infants with low birth weight	1 (1.92)	4 (8.33)	—	—
Incidence of adverse outcomes	4 (7.69)	15 (31.25)	9.001	<0.001

**Table 6:** Comparison of adverse reaction rates between two groups (*n* (%)).

Adverse reactions	Observation group *n* = 52	Control group *n* = 48	*χ* ^2^	*P*
Itching	1 (1.92)	2 (4.17)	—	—
Erythema	1 (1.92)	3 (6.25)	—	—
Temporary vaginal bleeding	0	3 (6.25)	—	—
Incidence of adverse reactions	2 (3.85)	8 (16.67)	4.558	0.033

## Data Availability

The labeled datasets used to support the findings of this study are available from the corresponding author upon request.
